The article "Three-Dimensional Finite Element Analysis of L4-5 Degenerative Lumbar Disc Traction under Different Pushing Heights" was published in 2021. Journal: J Healthc Eng.

# Three-Dimensional Finite Element Analysis of L4-5 Degenerative Lumbar Disc Traction under Different Pushing Heights

**DOI:** 10.1155/2021/1322397

**Published:** 2021-07-19

**Authors:** Huaili Ding, Lijun Liao, Peichun Yan, Xiaolin Zhao, Min Li

**Affiliations:** Fujian Maternity and Children's Hospital, Affiliated Hospital of Fujian Medical University/Fujian Children's Hospital, Fujian Fuzhou 350000, China

## Abstract

**Objective:**

To study and analyze the changes of intervertebral foramen height and area of the degenerative L4-5 intervertebral disc under different pushing heights by the finite element method.

**Methods:**

CT and MRI images of T12-S1 segments were obtained from a healthy volunteer who met the inclusion criteria. A DR machine was used to capture images of the lumbar lateral section before and after simultaneous pushing of the L4 and L5 spinous processes by manipulation called Daogaijinbei, and the measurement showed that the displacement changes of L4 and L5 were both approximately 10 cm, so the pushing height was set at 0–10 cm. A three-dimensional finite element model of the entire normal lumbar spine was established using Mimics 16.0, Geomagic Studio 2014, Hypermesh 13.0, MSC.Patran 2012, and so on. The disc height and nucleus area of the lumbar disc of the normal entire lumbar disc model were adjusted to establish models of the L4-5 disc with mild, moderate, and severe degeneration. Changes of disc height and area of the L4-5 degenerative intervertebral disc under different pushing heights were calculated.

**Results:**

The size of the L4-5 intervertebral foramen was analyzed from the height and area of the intervertebral foramen, and the results showed the following: (1) as for the normal lumbar disc and a lumbar of the L4-5 disc with mild and moderate degeneration, the height of the L4-5 intervertebral foramen and its area both increased during pushing between 0 and 8 cm. After the pushing height reached 8 cm, the height and area of the L4-5 intervertebral foramen gradually became stable; (2) as for the L4-5 disc with severe degeneration, during the process of pushing, the height and area of the L4-5 intervertebral foramen increased slightly, but this change was not obvious.

**Conclusions:**

After the spinal manipulation, the sizes of the L4-5 intervertebral foramen of the L4-5 disc with mild and moderate degeneration were significantly larger than those before pushing; in contrast, the size of L4-5 intervertebral foramen of the L4-5 disc with severe lumbar degeneration was not significantly changed.

## 1. Introduction

Lumbar intervertebral disc degeneration can cause biomechanical changes of the lumbar vertebrae and destroy their mechanical environment, thus resulting in a series of degenerative diseases of the lumbar intervertebral discs. Lumbar disc degeneration is a complex process in which the lumbar spine is affected by a variety of complex factors and changes in stroma composition or stroma state, and it is confluence by lumbar disc aging, biomechanical factors [1–3], nutritional factors [4–6], and so on. The main clinical manifestations of degenerative disease of the lumbar intervertebral discs are lumbago and leg pain, which are mainly caused by extrusion of a nerve root by protrusion after degeneration of the lumbar intervertebral disc. As lots of studies [7, 8] have showed, traditional Chinese massage therapy can effectively treat lumbar intervertebral disc degeneration. In this study, the relationship between the degree of L4-5 intervertebral disc degeneration and the corresponding intervertebral height and area was studied by the finite element analysis under different pushing heights of the traditional Chinese manipulation called Daogaijinbei.

The article "Three-Dimensional Finite Element Analysis of L4-5 Degenerative Lumbar Disc Traction under Different Pushing Heights" was published in 2021. Journal: J Healthc Eng.

## 2. Materials and Methods

### 2.1. Research Object

Creation of a three-dimensional finite element model of the whole normal lumbar and the models of the L4-5 disc with mild, moderate, and severe degeneration established based on CT and MRI images of the lumbar vertebrae of a healthy male volunteer, aged 26 years, with height 171 cm, weight 60.5 kg, no lumbar spinal stenosis, lumbar spondylolisthesis, or lumbar instability, and no ossification of intervertebral space, posterior longitudinal ligament, ligamentum flavum, vertebral anterior margin hyperplasia, and complex disease is not suitable for the study. The finite element method can simulate the material properties, morphological structure, boundary conditions, and load conditions of lumbar vertebrae in the digital form, observe any parameter that can change the influence on the mechanics of the entire lumbar vertebrae, and can be repeated loading and arbitrary testing. In addition, the research object referred to most literatures was 1 healthy adult, so the research object in this study was 1 healthy adult male volunteer.

### 2.2. Establishment of a Normal Full Lumbar Finite Element Model

In the imaging department of the affiliated rehabilitation hospital of Fujian University of Traditional Chinese Medicine, a healthy male volunteer was examined by CT imaging. Imaging examination and clinical confirmation showed that the volunteer was in good health, and his lumbar vertebrae were normal. The man voluntarily agreed to participate in the research subject and signed the informed consent form. The study passed the requirements of the hospital ethics committee. Images of the lumbar spine were acquired by CT scanning of T12-S1 segments using a Toshiba Aquilion 16 slice spiral CT, and MRI images were acquired using a Siemens 3.0 T MRI machine to continuously scan the lumbar spine. The scanning data were directly saved in a DICOM (digital imaging and communications in medicine) format. After completion of the lumbar CT and MRI image acquisition, Mimics 16.0, Geomagic Studio 2014, and Hypermesh 13.0 were used to complete the creation of a three-dimensional finite element model of the lumbar spine. After the model was established, MSC.Patran 2012 was used to calculate the size of the L4-5 intervertebral foramen under different pushing heights. Due to the complex range of motion of intervertebral joints, facet joints were not taken into account in this study, and the study was limited to the changes of intervertebral foramen.

The article "Three-Dimensional Finite Element Analysis of L4-5 Degenerative Lumbar Disc Traction under Different Pushing Heights" was published in 2021. Journal: J Healthc Eng.

The preprocessed CT images were imported into Mimics software, and the mask between the vertebrae was divided by edit masks. Then, the region growing tool was used to establish the vertebral lamina, and the vertebral model was generated from these laminas. Next, the model was filled with cavities and deburred using edit masks to obtain a model of the lumbar vertebrae with a smooth surface. Finally, a 3D model of the entire lumbar spine was generated using Calculate 3D, and the 3D model was postprocessed and meshed. Through the above steps, a finite element mesh model of the whole lumbar region was obtained as shown in Figure 1, and the mesh model of the intervertebral disc is shown in Figures 2 and 3.

Referring to the published literature [9–13], the parameter settings of L1-L5 lumbar vertebrae structural materials are given in Table 1.

## 3. Establishment of L4-5 Degenerative Disc Models

At present, there is no uniform standard for the specific grade of intervertebral disc degeneration. In this study, referring to the MRI grading standard of the Pfirrmann classification of intervertebral disc degeneration [14] (Table 2) and the Thompson five-level system [15], the process of intervertebral disc degeneration was considered from two aspects: disc height and nucleus pulposus area.

Classes I and II were categorized as a normal lumbar disc, III as mild degeneration, and IV and V as severe degeneration. On the basis of the effective normal three-dimensional finite element model, the degeneration of a lumbar intervertebral disc was simulated by reducing the height of the intervertebral disc and the area of the nucleus pulposus. The L4-5 intervertebral disc mild degeneration model was generated from the normal lumbar disc model by reducing the height by 15% while keeping the nucleus pulposus area unchanged, the moderate L4-5 intervertebral disc degeneration model was obtained by a 33% height reduction and a 67% nucleus pulposus area reduction, and the severe L4-5 intervertebral disc degeneration model was obtained by a 70% height reduction and a 67% nucleus pulposus area reduction.

The article "Three-Dimensional Finite Element Analysis of L4-5 Degenerative Lumbar Disc Traction under Different Pushing Heights" was published in 2021. Journal: J Healthc Eng.

Based on the above L4-5 intervertebral disc degeneration classification method, the parameters of the normal lumbar model were adjusted to establish whole lumbar models of mild, moderate, and severe degeneration of the L4-5 spine and of the L4-5 intervertebral disc, as shown in Figures 4–12.

### 3.1. Loading Mechanical Parameters

Lumbar vertebrae account for approximately 13.9% of human bodyweight [16]. The weight of the volunteer used for this model was 60.5 kg, making the weight of lumbar vertebrae approximately 8.41 kg, which is 84.1 N. Meanwhile, considering the pressure between other tissues, this study measured the waist pressure range of the doctor's palm on the subject's waist during the normal performance of lumbar extension with the help of a pressure sensor, and the maximum pressure was 99 N [17]. Thus, for convenience of calculation, the force applied to the L4 and L5 spinous processes was defined as 100 N in the finite element analysis.

The corresponding nodes on the upper surface of vertebral body L1 and the lower surface of vertebral body L5 are restrained by sliding support, and the displacement changes in flexion and extension directions are allowed, while different degrees of displacement are released. Considering the changes in the normal physiological curvature of the lumbar spine, the stress changes of the lumbar spine under different jacking heights were studied.The force is applied perpendicular to the spinous process nodes, and some nodes of L4 and L5 are constrained by releasing different displacement boundaries on the surfaces of L4 and L5 anterior longitudinal ligaments. The lateral sections of the lumbar spine before and after the action of the spinous process of L4 and L5 with the reverse cover were taken with a DR camera, respectively. The safe movement range of the spinous process of L4 and L5 was measured to be 10 cm. After the validity verification of the lumbar model, the mechanical parameters were loaded. The safe range of L4 and L5 lumbar vertebrae was within 10 cm, and the dynamic loading was carried out with 1 cm as the step length.The stress and distribution of each lumbar structure were observed. During the simulation calculation, the specific boundary constraint conditions of the spine manipulation bed simulating the inverted cover method on the whole lumbar spine are shown in Figure 13.

### 3.2. Calculation Method of Intervertebral Foramen Size

Research [18] shows that the maximum height and area of an intervertebral foramen decrease with the aggravation of intervertebral disc degeneration, while the maximum width of an intervertebral foramen is not affected by intervertebral disc degeneration, and that intervertebral disc degeneration is closely related to the height and area of the intervertebral foramen, and the calculation method used in the model established in this study is shown in Figure 14.

The article "Three-Dimensional Finite Element Analysis of L4-5 Degenerative Lumbar Disc Traction under Different Pushing Heights" was published in 2021. Journal: J Healthc Eng.

Using the method shown in the figure, we analyzed the changes in the lumbar structure when subjected to the stress of a normal L4-5 intervertebral disc and degenerative L4-5 discs with different degrees of degeneration, under different pushing heights of 0–10 cm. The size of the intervertebral foramen was measured and analyzed in the normal group, mild degeneration group, moderate degeneration group, and severe degeneration group.

## 4. Results

In the normal, mild degeneration, moderate degeneration, and severe degeneration groups, the L4 and L5 spinous processes were pushed up to a height of 0–10 cm, and the finite element experiment was conducted every 1 cm step. Considering that the L4-L5 structure is relatively symmetrical, the height and area of the intervertebral foramen on the one side were measured. As the results showed, the L4-5 intervertebral foramen heights of a normal lumbar disc and a lumbar of the L4-5 disc with mild and moderate degeneration were 20.1–25.9 mm, 18.4–24.9 mm, 14.5–20.2 mm, respectively, and the areas of the L4-5 intervertebral foramen were 235.2–341.9 mm^2^, 199.9–313.3 mm^2^, and 166.8–253.6 mm^2^, respectively. As for the L4-5 disc with severe degeneration, during the pushing process, the height of the L4-5 intervertebral foramen was 9.1–10.2 mm, and the area was 121.6–154.1 mm^2^. The changes during the pushing with different pushing heights are shown in Figure 15.

From Figure 15, the heights of the L4-5 intervertebral foramen and its areas of the normal lumbar disc and a lumbar of the L4-5 disc with mild and moderate degeneration both increased when the pushing height is between 0 and 8 cm, and the height and area of the L4-5 intervertebral foramen gradually became stable when the pushing height reached 8 cm or larger; however, the height and area of the L4-5 intervertebral foramen of the L4-5 disc with severe degeneration increased slightly, but this change was not obvious during the pushing.

## 5. Conclusions

After the spinal manipulation, the sizes of the L4-5 intervertebral foramen of the L4-5 disc with mild and moderate degeneration were significantly larger than those before pushing; in contrast, the size of L4-5 intervertebral foramen of the L4-5 disc with severe lumbar degeneration was not significantly changed.

The article "Three-Dimensional Finite Element Analysis of L4-5 Degenerative Lumbar Disc Traction under Different Pushing Heights" was published in 2021. Journal: J Healthc Eng.

## 6. Discussion

The size of the intervertebral foramen is closely related to the normal physiological morphology of spinal nerves and blood vessels, and some studies have shown that intervertebral disc degeneration is closely related to the height and area of the intervertebral foramen [19–22]. In this study, we analyzed the stress changes of the degenerative L4-5 intervertebral disc during pushing to a height of 0–10 cm and also analyzed the height and area of intervertebral foramen in these biomechanical environments. The height and area of the L4-5 foramen in mild, moderate, and severe degeneration of the L4-5 intervertebral disc were smaller than those of the normal lumbar spine when the pushing height was 0 cm, i.e., with no pushing. The height and area of the L4-5 intervertebral foramen decreased with increased L4-5 intervertebral disc degeneration. For the lumbar vertebrae with mild and moderate degeneration of the L4-5 intervertebral disc, the height and area of the L4-5 intervertebral foramen showed a continuously increasing trend when the pushing height was 0–8 cm. When the pushing height was 8–10 cm, the height and area of the L4-5 intervertebral foramen gradually became stable, which indicated that the height and area of the L4-5 intervertebral foramen of mild and moderate degeneration of the L4-5 intervertebral disc could be improved under spinal manipulation, and the height and area of the L4-5 intervertebral foramen tended to remain stable after the pushing height reached 8 cm. For the L4-5 intervertebral disc with severe degeneration, the height and area of L4-5 intervertebral foramen did not increase significantly; therefore, the pushing effect of spinal manipulation did not have a significant effect on the size of the L4-5 intervertebral foramen [23, 24].

## Figures and Tables

**Figure 1:** The finite element mesh model of the whole lumbar spine.

**Figure 2:** Whole lumbar disc mesh model.

**Figure 3:** Whole lumbar disc mesh model.

**Figure 4:** Lumbar model of L4-5 disc mild degeneration.

**Figure 5:** Whole disc model of L4-5 disc mild degeneration.

**Figure 6:** L4-5 disc model with mild.

**Figure 7:** Lumbar model of L4-5 disc moderate degeneration.

**Figure 8:** Whole disc model of L4-5 disc moderate degeneration.

**Figure 9:** L4-5 disc model with moderate degeneration.

**Figure 10:** Lumbar model of L4-5 disc severe degeneration.

**Figure 11:** Whole disc model of L4-5 disc severe degeneration.

**Figure 12:** L4-5 disc model with severe degeneration.

**Figure 13:** Boundary constraint conditions of the whole lumbar spine.

The article "Three-Dimensional Finite Element Analysis of L4-5 Degenerative Lumbar Disc Traction under Different Pushing Heights" was published in 2021. Journal: J Healthc Eng.

**Figure 14:** Measurement of intervertebral foramen morphology (height, width, and area) (AB is the height of the intervertebral foramen, CD is the width of the intervertebral foramen, and E is the area around ABCD, the area of the intervertebral foramen).

**Figure 15:** The (a) height and (b) area of L4-5 intervertebral foramen under different pushing heights.

**Table 1:** Structural material parameters of L1-L5 lumbar spine.

Structure	Modulus of elasticity (MPa)	Poisson's ratio
Cortical bone	12000	0.30
Cancellous bone	100	0.20
Endplate	2000	0.20
Back-end structure	3500	0.30
Annulus fibrosus	92	0.45
Annulus fibrosus matrix	4.2	0.45
Nucleus pulposus	1.0	0.499
Anterior longitudinal ligament	7.8	0.30
Posterior longitudinal ligament	10	0.30
Supraspinous/interspinous ligaments	8	0.30
Cystic ligament	15	0.30
Ligamentum flavum	10	0.30
Intertransverse ligament	10	0.30
Facet joint	10	0.30

**Table 2:** Pfirrmann classification.

Grade	Nucleus pulposus structure	Boundaries of nucleus pulposus and annulus fibrosus	Nucleus pulposus signal intensity	Disc height
I	Uniform, bright white	Clear	High	Normal

II	Uneven, may have horizontal zone	Clear	High	Normal

III	Uneven, gray	Not clear	Medium	Slightly reduced

IV	Uneven, gray to black	Loss	Medium to low	Moderately reduced

V	Uneven, black	Loss	Low	Severely reduced

## Data Availability

The data used to support the findings of this study cannot be shared as no datasets were generated or analyzed during the current study.
